# Characteristics of a water-forming NADH oxidase from *Methanobrevibacter smithii*, an archaeon in the human gut

**DOI:** 10.1042/BSR20160357

**Published:** 2016-11-17

**Authors:** Mingguang Yan, Weibing Yin, Xiao Fang, Jianjun Guo, Hong Shi

**Affiliations:** * Department of Clinical Laboratory, The First People's Hospital of Shangqiu City, Shangqiu 476000, China; † Department of Infectious Diseases, The Third Affiliated Hospital of Sun Yat-Sen University, Guangzhou 510630, China

**Keywords:** enzyme kinetics, *Methanobrevibacter smithii*, NADH oxidase, protein function

## Abstract

NADH oxidases (NOXs) catalysing the oxidation of NADH to yield NAD^+^ and H_2_O, H_2_O_2_, or both play an important role in protecting organisms from oxidative stress and maintaining the balance of NAD^+^/NADH. A gene encoding NOX was identified from *Methanobrevibacter smithii* (NOX-ms), the predominant archaeon in the human gut ecosystem. Subsequent analyses showed that it is an FAD-containing protein with a subunit molecular mass of 48 kDa. NOX-ms was purified to homogeneity after expression in *Escherichia coli*. NOX-ms catalysed the oxidization of NADH and converted O_2_ to H_2_O with an optimal pH of 7.5 and a temperature optimum of approximately 37°C. The *V*_max_ and *K*_m_ values were 42.6–44.1 unit/mg and 47.8–54.6 μM for NADH. The apparent *V*_max_ and *K*_m_ for oxygen were 189.5–196.1 unit/mg and 14.6–16.8 μM. The mutation analysis suggests that Cys^42^ in NOX-ms plays a key role in the four-electron reduction of O_2_ to H_2_O. Quantitative reverse transcription-PCR (RT-qPCR) revealed that transcription of *NOX-ms* was also up-regulated after exposing the cells to oxidative stress and glucose. Finally, the potential of NOX-ms as a target to control colonization of *M. smithii* and its possible applications are discussed.

## Abstract (precis)

NOX-ms catalysed the oxidization of NADH and converted O_2_ to H_2_O by using cysteine-mediated electron transfer. Its transcription was increased by oxidative stress and glucose.

## INTRODUCTION

Recently, a role of the gut microbiota has been attracting more attention. Besides the many bacterial species, the human gut contains several archaeal species but only three distinct species within the group of methanogenic archaea have been isolated from human faeces, *Methanobrevibacter smithii* [1], *Methanosphaera stadtmanae* [2] and *Methanomassilicoccus luminyesis* [3]. *M. smithii* belonging to the *Methanobacteriaceae* family is the dominant archaeon in the human gut ecosystem [4]. In children from 1 to 10 years of age, the prevalence of *M. smithii* has been found in 88% [5]. This organism plays an important role in the efficient digestion of polysaccharides (complex sugars) by consuming the end products of bacterial fermentation [6]. Metagenomics studies of the gut microbial communities in genetically obese mice have shown that *M. smithii* exhibited an enhanced expression of the genes involved in polysaccharide degradation and possess a greater capacity to promote adiposity when transplanted into germ-free recipients [4]. A recent research showed that *M. smithii* colonization was associated with an increased risk of overweight children from 6 to 10 years of age [7]. *M. smithii* may thus be a therapeutic target for childhood overweight and obesity by reducing energy harvesting.

NADH oxidase (NOX) is a member of the flavoprotein disulfide reductase family that catalyses the pyridine-nucleotide-dependent reduction of various substrates, including O_2_, H_2_O_2_ and thioredoxin [8]. There are two types of NOXs that are H_2_O_2_-forming (NOX-1) and H_2_O-forming (NOX-2) respectively. NOX-1 catalyses the two-electron reduction of O_2_ to H_2_O_2_ by NADH, whereas NOX-2 catalyses the four-electron reduction of O_2_ to H_2_O by NADH [8]. The deduced amino acid sequences between the NOX-1 and NOX-2 showed low homology [9,10]. NOXs play diverse physiological roles, depending on its substrates and products in different organisms. NOX-1 is part of an alkyl hydroperoxide reductase system *in vivo* in combination with alkyl hydroperoxide reductase subunit C in *Amphibacillus xylanus* and *Streptococcus mutans* [11,12]. NOX-1 from thermophilic *Archaeoglobus fulgidus* may be involved in electron transfer in sulfate respiration [13]. NOX-2 are considered to be important enzymes in protecting against oxidative stress through their capacity to reduce O_2_ to H_2_O without the formation of harmful reactive oxygen species [14] and in regenerating NAD^+^ during aerobic mannitol metabolism, acts an important role in aerobic energy metabolism in O_2_-tolerant *Streptococcus mutans* and maintaining the balance of NAD^+^/NADH [11]. In application, some of the NOX-2 were successfully applied to control the level of intracellular cofactors to redirect cellular metabolism [15–18].

Despite the importance of NOX in protecting against oxidative stress and energy metabolism, little is known about the function of NOX in *M. smithii*. In the present study, a water-forming NOX was identified from *M. smithii*. The recombinant His-tag NOX from *M. smithii* (NOX-ms) was efficiently produced in a bacterial expression system and purified by immobilized metal affinity chromatography. Afterward, the enzyme was biochemically characterized and used mutants to analyse the catalytic mechanism. The expression level of NOX-ms under different conditions was finally analysed.

## MATERIALS AND METHODS

### Protein expression and purification

*M. smithii* strain PS (ATCC 35061) was cultivated in 125 ml serum bottles containing 15 ml of *Methanobrevibacter* complex medium supplemented with 3 g/l formate, 3 g/l acetate and 0.3 ml of a freshly prepared, anaerobic, filter-sterilized 2.5% Na_2_S solution. The remaining volume in the bottle (headspace) contained a 4:1 mixture of H_2_ and CO_2_; the headspace was replenished every 1–2 d during a 6-d growth period at 37°C. DNA was recovered from harvested cell pellets using the Qiagen Genomic DNA Isolation kit, with mutanolysin (1 unit/mg wet-weight cell pellet; Sigma) added to facilitate microbe lysis.

*M. smithii* genomic DNA was used as a template in a PCR, which isolated *NOX-ms* (Msm_0046, WP_004033913) using the following oligonucleotide primers: forward, 5′-CG G AATTC ATG AAA GTT GTT ATT G-3′ and reverse, 5′-CCG CTCGAG TTA GTT AAA TTT CTT AC-3′. The primers introduce restriction sites EcoRI and XhoI (underlined) respectively. PCR products were ligated into the pET28 (a) vector and sequenced before transformation into BL21 (DE3). *Escherichia coli* BL21 (DE3) cells containing the *pET28-NOX-ms* plasmid were cultured. When the *A*_600_ reached 0.7, IPTG was added to induce protein expression. The cells were cultured in the presence of IPTG for 4 h with shaking and then harvested and resuspended in lysis buffer containing 50 mM Tris (pH 8.0), 300 mM NaCl, 20 mM 2-mercaptoethanol and 20 mM imidazole. The cell suspension was sonicated and centrifuged at 20000 ***g*** for min, and the supernatant was loaded on a Ni-NTA column. After washing the column with lysis buffer, NOX-ms was eluted using an imidazole gradient (50–250 mM). Purified protein was separated on a SDS/10% PAGE and visualized. Protein concentrations were estimated using the Bradford method and BSA as a standard [19].

### Site-directed mutagenesis of NOX-ms

The primers used for the single cysteine to serine mutant (underlined) were as follows: Cys^42^, forward, 5′-TAT TCT CCA GCT GCT ATT CCT-3′; reverse, 5′-AGG AAT AGC AGC TGG AGA ATA-3′; Cys^230^, forward, 5′-GAC GGA AGC GCT ATT GAT GCA-3′; reverse, 5′-TGC ATC AAT AGC GCT TCC GTC-3′. The pET28a-NOX-ms plasmid was used as the DNA template. The PCR reaction was performed for 18 cycles (94°C for 30 s, 55°C for 1 min and 68°C for 12 min). After amplification, the PCR mixture was digested with DpnI and used to transform *E. coli* BL21(DE3). The mutant was confirmed by DNA sequencing. The NOX-ms-C42A and NOX-ms-C230A were purified by the same methods as that of the wild-type protein, as described above.

#### Spectra analysis of NOX-ms and Apo-NOX-ms preparation

The purified enzymes were scanned in the air-saturated 100 mM sodium phosphate buffer (pH 7.0) at room temperature in a 1.0 ml quartz cuvette. The absorption spectrum (300–800 nm) was recorded in the spectrophotometer.

The purified NOX-ms from *E. coli* is a holoenzyme with FAD. The protein was dialysed with 100 mM phosphate buffer (pH 7.2) containing 2.4 M (NH_4_)_2_SO_4_, 20 mM 2-mercaptoethanol and 0.5 mM EDTA, and then loaded on the hydrophobic interaction chromatography column equilibrated with the same buffer. FAD was eluted with equilibration buffer saturated with NaBr (pH 3.5). The column was balanced again with the equilibration buffer, and the apoprotein was eluted with 100 mM phosphate buffer.

### Assays for NOX-ms activity

The NOX activity of the recombinant protein was examined by time-dependent removal of NADH in aerobic conditions. The assays were performed in 50 mM sodium phosphate buffer (pH 7.2), 0.5 mM NADH or NADPH and 100 mM NaCl at the indicated temperatures. The reaction was started by adding NOX-ms in the amounts indicated. The rate of NADH consumption was measured by monitoring the decrease in *A*_340_ in a UV–visible spectrophotometer (INESA Instrument). One unit of activity was defined as the amount of enzyme catalysing the oxidation of 1 μmol NADH or O_2_ per min at 37°C in 50 mM sodium phosphate buffer (pH 7.2).

For kinetic studies, the initial velocities of the enzymatic reaction were examined by varying the concentration of NADH (from 0.02 to 0.6 mM) in the optimal conditions. For the O_2_ monitor assay, NOX activity was measured using an anaerobic glass cuvette in 50 mM potassium phosphate buffer (pH 7.0) inflating with different concentration of oxygen. The reaction was started by the addition of enzyme solution, and the decrease in oxygen concentration was monitored with a Clark-type oxygen electrode (Rex Electric, JPB-607A). Values of the *Michaelis* constants (*K*_m_) and maximal velocity (*V*_max_) were obtained by mathematical calculations according to SigmaPlot software. The parameters were determined by three separate experiments.

### Quantification of H_2_O_2_

NOX assay mixtures containing various concentrations of NADH (0.1–0.5 mM) were incubated at 37°C and the reaction was allowed to go to completion. The solution (250 μl) was combined with 50 μl of a solution containing Amples Red and 100 unit/ml horseradish peroxidase (Aladdin). After incubation at room temperature for 30 min, the absorbance at 560 nm was measured. The amount of H_2_O_2_ produced in the assay was determined according to the absorbance value and a standard curve.

### Quantitative reverse transcription-PCR)

The culture of *M. smithii* was carried out in as described above. The cells were shocked by exposure to oxygen (1–8% O_2_ was sparged into the growth environment) or in the presence of glucose (1–4 g/l) and incubating for 6 h. Survival of the cells was estimated by the three-tube most probable number method after exposure to stress. The cells were harvested and RNA was prepared with TRIzol reagent (Invitrogen). To ensure complete removal of any contaminating DNA, all RNA preparations were given a DNAase treatment (Thermo Scientific Fermentas). RNA was quantified with a spectrophotometer and cDNA was synthesized with the Universal RiboClone cDNA Synthesis System (Promega) according to the manufacturer's protocols. The reaction products were serially diluted to find the adequate concentration for real-time PCR analysis using the following primers: 5′-GGT GAC GGA AGC TGT ATT GA-3′ and 5′-AGC CCA TCT TCC GAT ATC AC-3′. Real-time PCR was performed in CFX96 Real-Time PCR System (Bio–Rad Laboratories), using SYBR Green PCR Master Mix (Toyobo, Japan). The relative fold changes were determined from cycle threshold (*C*_T_) values using the ΔΔ*C*_T_ method. The reactions for detection of 16S rRNA (Msm_1801) levels were used for normalization between the different samples, which were amplified with primers: 5′-CTG CAG CTT AAC TGT GGG AA-3′ and 5′-GGT CCT CCC AGG ATT ACA GA-3′. The experiments were analysed in three independent assays, with at least three technical replicates included in each PCR to ensure reproducibility.

## RESULTS

### Sequence analysis of NOX-ms

Homology and domain search of the *M. smithii* genome identified a homolog of NOX (*NOX-ms*, Msm_0046) that was not characterized before. Sequence analysis revealed that *nox-ms* encodes a protein of 444 amino acids, with a theoretical pI of 4.8 and a theoretical molecular mass of 48.180. A BLAST-P search in National Center for Biotechnology Information (NCBI) for the NOX-ms sequence revealed the most significant homology (35–64% identity) with the proteins from methanogenic archaea (*Methanothermobacter thermoautotrophicus*, *Methanocaldococcus jannaschii*). NOX-ms also showed >30% identity to the proteins from other archaea (*Thermococcus kodakarensis*, *Pyrococcus abyssi*), bacteria (*Halonatronum saccharophilum*, *Hydrogenibacillus schlegelii etc.*) and eukaryotes (*Cladophialophora immunda*, *Exophiala oligosperma*, *Metarhizium anisopliae*, *etc.*). To explore the evolutionary relationship between NOX-ms and other annotated NOXs, the MEGA6 program was used to construct a phylogenetic tree from amino acid sequence data. Although the bootstrap values were somewhat low because of a large number of sequences, more significant bootstrap values in the distal branches allowed us to infer those proteins from similar species that were derived from a common ancestor. Furthermore, their positions in the dendrogram were independent of the method used for phylogenetic reconstruction (results not shown).

The amino acid composition of NOX-ms revealed the presence of eight cysteine residues and multiple sequence alignment (Figure 1B) revealed that Cys^42^ is located at a similar position to that of the cysteine residue in the conserved active site of other NOXs. The conserved motifs were also identified in the amino acids sequence alignment. One was an FAD-binding domain containing the AMP-binding and FMN-binding motifs observed in enzymes belonging to the glutathione reductase family. The other domain was a glycine-rich NAD-binding motif located between the AMP-binding and FMN-binding motifs (two FAD-binding domains) [20].

**Figure 1:** Phylogenetic and sequence analysis of NOX-ms and other NOXs (**A**) Molecular phylogenetic analysis of NOXs from archaea (green), bacteria (blue) and eukarya (orange) by Maximum Likelihood method generated using MEGA6. The evolutionary history was inferred by using the Maximum Likelihood method based on the Jones-Taylor-Thornton matrix-based model. The tree with the highest log likelihood (−10270.1967) is shown. The percentage of trees in which the associated taxa clustered together is shown next to the branches. The percentage of replicate trees in which the associated taxa clustered together in the bootstrap test (1000 replicates) is shown next to the branches. The accession numbers of the proteins are indicated after the names’ of the species. (**B**) Sequence alignment of NOX-ms and other homologues. The residues involved in FAD binding are labelled in solid lines. The NAD-binding site is highlighted by a dash line. The active site of cysteine is labelled by a star. The shading indicates residues that are identical and the boxed amino acids represent positions with a lower level of conservation.

### Purification of NOX-ms and apo-NOX-ms preparation

In order to understand the function of NOX-ms, the *nox-ms* gene was successfully amplified from genomic *M. smithii* DNA and cloned to plasmids adding a His-Tag at' the N-terminus. The purification of recombinant NOX-ms from *E. coli* was performed by affinity chromatography as described in section ‘Materials and methods’. SDS/PAGE analysis of recombinant NOX-ms revealed a molecular mass of approximately 50 kDa (Figure 2A). Meanwhile, the enzymes with N-terminal His-Tag were soluble and could be purified as a yellowish solution due to the bound FAD, because the isoalloxazine ring system in FAD can induce light absorbance in the UV and visible spectral range, giving rise to the yellow appearance of flavin and flavoproteins. Purified NOX-ms from *E. coli* has absorption maxima at 378 nm and 456 nm, with a shoulder at 480 nm, which is characteristic spectral feature of proteins with bound flavin cofactors. As NOX-ms contains FAD as a prosthetic group, apo-NOX-ms was prepared by hydrophobic interaction chromatography under acidic conditions (pH 3.5) with saturated NaBr buffer [21], in order to confirm the function of FAD. The absorption spectrum of apo-NOX-ms did not show any significant absorbance in the visible region, revealing that FAD was indeed absent (Figure 2B). The holoenzyme can be reconstituted by incubating equimolar concentrations of apomonomers and FAD at room temperature for 5 min. After dialysis to remove unbinding FAD, the absorbance of the enzyme can be recovered. Compared the absorbance of the native enzyme and reconstituted enzyme, the absence of an absorbance feature in the 480 nm region of the reconstituted enzyme were observed. A similar lack of absorbance shoulder in this region is seen in spectra reported in previous studies of NOX [22] and other flavoproteins [23], implicating that the protein may have lower affinity to cofactors than the native protein [24].

**Figure 2:** Purification and spectra of NOX-ms (**A**) Purification of NOX-ms. Proteins were electrophoresed on a 12.5% SDS-polyacrylamide gel and stained with Coomassie brilliant blue G-250. Lane M, protein marker; the molecular mass standards are indicated at the left. (**B**) Spectra of NOX-ms (solid line), apo-NOX-ms (dotted line) and the reconstituted NOX-ms (dash line). The absorbance was measured in 50 mM sodium phosphate buffer (pH 7.2) at room temperature with the protein concentration of 0.5 mg/ml.

### Catalytic characterization of NOX-ms

NOXs from *Lactobacillus sanfranciscensis* [25], *Pyrococcus horikoshii* [26] and *Thermococcus profundus* [22] accept both NADH and NADPH as cofactors. The NOX and NADPH oxidase activity of NOX-ms was also measured. The assays revealed that NOX-ms preferred NADH as the active substrate, and the activity towards NADPH was approximately 20% of that to NADH (Supplementary Figure S1). In the further research, NADH was used as the reducing substrate to determine the function of NOX-ms. In the temperature activity experiments, the NOX activity of NOX-ms was measured at temperatures ranging from 25°C–50°C at a constant pH of 7.2. The results revealed that the optimum temperature for the enzyme was approximately 37°C (Figure 3A). To study the effect of pH, the NOX activity of the purified enzyme were surveyed between pH values of 5.0 and 10.0 at an assay temperature of 37°C. The pH profile of the purified NOX-ms is shown in Figure 3(B). The enzyme was most active between pH values 6.5–8.0, with maximal activity at pH 7.5. The kinetics of recombinant NOX-ms were analysed using NADH as a substrate by varying its concentration. The Michaelis–Menten equation was used to calculate the kinetic parameters (Figure 3B). NOX-ms could catalyse NADH oxidization with an apparent *K*_m_=47.8–54.6 μM and *V*_max_=42.6–44.1 unit/mg (*n*=9). The kinetic parameters for O_2_ was also measured by varying O_2_ concentration and keeping NADH concentration to be constant, which showed that NOX-ms could remove O_2_ with an apparent *K*_m_=14.6–16.8 μM and *V*_max_=189.5–196.1 unit/mg (*n*=9).

**Figure 3:** Enzyme activity assays of NOX-ms (**A**) Optimal temperature of NOX-ms activity. (**B**) Optimal pH of NOX-ms activity. Different buffers were used for the different pH solutions used in this assay. MES buffer was used for pH 5.0 and 7.5; HEPES buffer was used for pH 8.0 and 8.5; glycine buffer was used for pH 9.0 and 10.0. (**C**) Kinetics assay of NOX-ms. (**a**) The velocity data changed with the increase in NADH concentrations were fitted to the Michaelis–Menten equation by non-linear regression calculations. (**b**) Effects of O_2_ on the velocity of the NOX of NOX-ms. The velocity data were fitted to the Michaelis–Menten equation by non-linear regression calculations. (**D**) Relative activity of wild-type NOX-ms, apo-NOX-ms, reconstituted NOX-ms, NOX-ms-C42A and NOX-ms-C230A with NADH as substrates. All experiments were performed in triplicate. The error bars mean the S.D. of three measurements.

To determine whether flavin cofactors were required for the enzymatic activity of NOX-ms, FMN, FAD and riboflavin were added as equimolar concentrations of apomonomers of holo-NOX-ms and the activity was measured. The results showed that external flavin cofactors have no significant effect on the activity (Supplementary Figure S2A). To further confirm the function of flavin cofactors, holo-enzyme and apo-enzyme activities were assayed. The activity of the reconstituted enzyme by FAD was also measured. These assays revealed that FAD significantly restored the oxidase activity of apo-NOX-ms (Figure 3D). Addition of other flavin cofactors such as FMN and riboflavin to apo-enzyme could not recover the enzyme activity. These results clearly indicated that NOX-ms is an FAD-dependent NOX.

Previous study showed that cysteine may function as the non-flavin redox centre in NOX [22]. The sequence alignment of NOXs (Figure 1B) revealed that NOX-ms contains eight cysteine residues and Cys^42^ may be the active site. As cysteines are important residues for NOX enzyme activity, we replaced Cys^42^ with alanine to analyse the function of the two residues. Cys^230^ was also mutated as a control. After purification using the same method as that used for the wild-type enzyme, NOX assays were performed with the two mutants under the same conditions as used for the wild-type. The results showed that the C230A mutant had similar NOX activity to that of the wild-type protein; however, the C42A mutant had <10% of the NOX activity of the wild-type protein (Figure 3D). Considering these results, Cys^42^ may provide the essential second redox centre in addition to the flavin.

Due to a conserved cysteine residue at position 42, NOX-ms should be an H_2_O-forming NOX. In order to determine the product of the NOX activity of NOX-ms, H_2_O_2_ was quantified using the Amples Red and horseradish peroxidase method [17]. The results demonstrated that less than 1% of the theoretical yield of hydrogen peroxide could be detected.

### The expression of *nox-ms* gene

As NOX may have a key role in oxidative stress tolerance [27] and sugar metabolism [18], gene expression level was studied by quantitative reverse transcription-PCR (RT-qPCR) to investigate the physiological role of NOX-ms. RNA was isolated from *M. smithii* cells grown under different concentration of oxygen. The results showed that there were no significant differences in the frequency of viable cells compared with control (Supplementary Figure S1). The relative expression patterns of *nox-ms* are shown in Figure 4. The lowest transcription level could be seen under anaerobic conditions. With increase in oxygen concentration, the expression level increased. Expression of *nox-ms* was also up-regulated by glucose in the media. Therefore, the physiological function of NOX-ms seemed to be related to both oxidative stress tolerance and sugar metabolism.

**Figure 4:** Expression level of *nox-ms* gene under oxidative stress and in the presence of glucose (**A**) The mRNA relative quantity of *nox-ms* under oxygen stress. *M. smithii* cells were treated by different concentration of oxygen (sparging 1–8% O_2_ into the growth environment) and the expression level of *nox-ms* was measured by RT-qPCR and indicated as fold difference from the value of the cells growing anaerobically, which is taken as 1. (**B**) The mRNA relative quantity of *nox-ms* from *M. smithii* cells growing in the presence of glucose. One to four grams per litre glucose were added in the media respectively and the expression level of *nox-ms* was measured by RT-qPCR and indicated as fold difference from the value of the cells growing without glucose, which is taken as 1. Error bars indicate the S.D. from three independent experiments (*P<0.05 and **P<0.01).

## DISCUSSION

*M. smithii* is the leading representative species in healthy volunteers [28] and plays a central role in the regulation of gut redox [29]. NOX is the key enzyme maintaining the redox balance in bacteria, plants and mammalians [30–32]. In addition, the biotechnological applications of NOXs as the regenerating system in redox reactions have been recently highlighted [33]. By the potential importance of the enzyme in *M. smithii*, a deeper understanding of its function is highly desirable. In the present study, we have demonstrated NOX-ms can efficiently reduce O_2_ to produce H_2_O using NADH as an electron donor. In addition, the activity assays of the wild-type, apo-enzyme and mutants showed that NOX-ms is an FAD-dependent enzyme and Cys^42^ is the active site residue. These results indicate that both FAD and Cys^42^ participate in the direct four-electron transfer reduction of O_2_ to H_2_O. Furthermore, the transcription level of NOX-ms was up-regulated under aerobic conditions and by glucose. Considering NOX-ms is involved in sugar metabolism and the relationship between *M. smithii* and overweight, we propose that NOX-ms can be a potential target to control the colonization of *M. smithii*.

H_2_O-forming NOXs in facultative anaerobes play an important role in the oxygen tolerance of these bacteria [8,34]. For example, mutants of *Streptococcus pyogenes* (facultative anaerobe) and *Brachyspira hyodysenteriae* (an aerotolerant anaerobe) with H_2_O-forming NOX-deficiency are unable to grow under high-O_2_ conditions, indicating the importance of NOX-scavenging activity against harmful O_2_ [34,35]. In *Clostridium aminovalericum*, an obligate anaerobe, H_2_O-forming NOX also exists as an oxygen-detoxifying enzyme [36]. In archaea, NOX from *Pyrococcus furiosus* produces both H_2_O_2_ (77%) and H_2_O (23%) [37] and NOX from *T. profundus* can catalyse electron transfer from NADH and NADPH to O_2_ and predominantly produce H_2_O [22]. NOX-ms only made H_2_O during its reaction with NADH and O_2_. The *V*_max_ value to O_2_ is approximately four times higher than that to NADH. The *K*_m_ to O_2_ is much lower than the value to NADH, implicating NOX-ms has much higher affinity to O_2_. The *K*_m_ value to O_2_ is also lower than the value (61.9 μM) of the enzyme from *C. aminovalericum* [36]. Meanwhile, the expression of NOX-ms was up-regulated by oxygen. We, therefore, propose that NOX-ms may decompose O_2_ and protect *M. smithii* from oxidative stress.

Lots of the oxidation reactions need the expensive cofactor, NAD^+^. At present, several processes have been applied to overcome cofactor regeneration, such as co-immobilization of bi-enzyme cascades on porous supports [38], engineering of glycerol dehydrogenase for regeneration of N6-CM-NAD^+^ [39] and simultaneous expression of two or more enzymes in a single cell [40]. One promising approach to regenerate NAD^+^ pools is the use of NOXs that reduce oxygen to hydrogen peroxide while oxidizing NADH to NAD^+^ [41]. Several NOXs from *Thermus thermophiles* [42], *Lactobacillus pentosus* [17] and *Bacillus subtilis* [43] have been reported to be used as the cofactor regeneration enzymes. On the other hand, NOX-ms was up-regulated by glucose, implicating that NOX-ms would utilize the glycolytic NADH to produce NAD^+^. Considering the advantage of producing water, NOX-ms has also the potential application in NAD^+^ regeneration.

## Abbreviations

NOX: NADH oxidase
RT-qPCR: quantitative reverse transcription-PCR

## References

[1] Miller T.L., Wolin M.J., Conway de Macario E., Macario A.J. (1982). Isolation of *Methanobrevibacter*
*smithii* from human feces. Appl. Environ. Microbiol..

[2] Miller T.L., Wolin M.J. (1985). *Methanosphaera stadtmaniae* gen. nov., sp. nov.: a species that forms methane by reducing methanol with hydrogen. Arch. Microbiol..

[3] Dridi B., Fardeau M.L., Ollivier B., Raoult D., Drancourt M. (2012). *Methanomassiliicoccus*
*luminyensis* gen. nov., sp. nov., a methanogenic archaeon isolated from human faeces. Int. J. Syst. Evol. Microbiol..

[4] Samuel B.S., Hansen E.E., Manchester J.K., Coutinho P.M., Henrissat B., Fulton R., Latreille P., Kim K., Wilson R.K., Gordon J.I. (2007). Genomic and metabolic adaptations of *Methanobrevibacter*
*smithii* to the human gut. Proc. Natl. Acad. Sci. U.S.A..

[5] Dridi B., Henry M., Richet H., Raoult D., Drancourt M. (2012). Age-related prevalence of *Methanomassiliicoccus*
*luminyensis* in the human gut microbiome. APMIS.

[6] Krajmalnik-Brown R., Ilhan Z.-E., Kang D.-W., DiBaise J.K. (2012). Effects of gut microbes on nutrient absorption and energy regulation. Nutr. Clin. Pract..

[7] Mbakwa C.A., Penders J., Savelkoul P.H., Thijs C., Dagnelie P.C., Mommers M., Arts I.C. (2015). Gut colonization with *Methanobrevibacter*
*smithii* is associated with childhood weight development. Obesity.

[8] Argyrou A., Blanchard J.S. (2004). Flavoprotein disulfide reductases: advances in chemistry and function. Prog. Nucleic Acid Res. Mol. Biol..

[9] Higuchi M., Shimada M., Matsumoto J., Yamamoto Y., Rhaman A., Kamio Y. (1994). Molecular cloning and sequence analysis of the gene encoding the H_2_O_2_-forming NADH oxidase from *Streptococcus*
*mutans*. Biosci. Biotechnol. Biochem..

[10] Matsumoto J., Higuchi M., Shimada M., Yamamoto Y., Kamio Y. (1996). Molecular cloning and sequence analysis of the gene encoding the H_2_O-forming NADH oxidase from *Streptococcus*
*mutans*. Biosci. Biotechnol. Biochem..

[11] Higuchi M., Yamamoto Y., Poole L.B., Shimada M., Sato Y., Takahashi N., Kamio Y. (1999). Functions of two types of NADH oxidases in energy metabolism and oxidative stress of *Streptococcus*
*mutans*. J. Bacteriol..

[12] Niimura Y., Nishiyama Y., Saito D., Tsuji H., Hidaka M., Miyaji T., Watanabe T., Massey V. (2000). A hydrogen peroxide-forming NADH oxidase that functions as an alkyl hydroperoxide reductase in Amphibacillus xylanus. J. Bacteriol..

[13] Reed D.W., Millstein J., Hartzell P.L. (2001). H_2_O_2_-forming NADH oxidase with diaphorase (cytochrome) activity from *Archaeoglobus*
*fulgidus*. J. Bacteriol..

[14] Miyoshi A., Rochat T., Gratadoux J.J., Le Loir Y., Oliveira S.C., Langella P., Azevedo V. (2003). Oxidative stress in *Lactococcus*
*lactis*. Genet. Mol. Res..

[15] Ji X.J., Xia Z.F., Fu N.H., Nie Z.K., Shen M.Q., Tian Q.Q., Huang H. (2013). Cofactor engineering through heterologous expression of an NADH oxidase and its impact on metabolic flux redistribution in *Klebsiella*
*pneumoniae*. Biotechnol. Biofuels.

[16] Kim J.W., Seo S.O., Zhang G.C., Jin Y.S., Seo J.H. (2015). Expression of *Lactococcus*
*lactis* NADH oxidase increases 2,3-butanediol production in Pdc-deficient *Saccharomyces*
*cerevisiae*. Bioresour. Technol..

[17] Zhang J.D., Cui Z.M., Fan X.J., Wu H.L., Chang H.H. (2016). Cloning and characterization of two distinct water-forming NADH oxidases from *Lactobacillus*
*pentosus* for the regeneration of NAD. Bioprocess Biosyst. Eng..

[18] Fang B., Jiang W., Zhou Q., Wang S. (2015). Codon-optimized NADH oxidase gene expression and gene fusion with glycerol dehydrogenase for bienzyme system with cofactor regeneration. PLoS One.

[19] Bradford M.M. (1976). A rapid and sensitive method for the quantitation of microgram quantities of protein utilizing the principle of protein-dye binding. Anal. Biochem..

[20] Dym O., Eisenberg D. (2001). Sequence-structure analysis of FAD-containing proteins. Protein Sci..

[21] Hefti M.H., Vervoort J., van Berkel W.J. (2003). Deflavination and reconstitution of flavoproteins. FEBS J..

[22] Jia B., Park S.C., Lee S., Pham B.P., Yu R., Le T.L., Han S.W., Yang J.K., Choi M.S., Baumeister W. (2008). Hexameric ring structure of a thermophilic archaeon NADH oxidase that produces predominantly H_2_O. FEBS J..

[23] Jackson R.G., Rylott E.L., Fournier D., Hawari J., Bruce N.C. (2007). Exploring the biochemical properties and remediation applications of the unusual explosive-degrading P450 system XplA/B. Proc. Natl. Acad. Sci. U.S.A..

[24] Bui S.H., McLean K.J., Cheesman M.R., Bradley J.M., Rigby S.E., Levy C.W., Leys D., Munro A.W. (2012). Unusual spectroscopic and ligand binding properties of the cytochrome P450-flavodoxin fusion enzyme XplA. J. Biol. Chem..

[25] Lountos G.T., Jiang R., Wellborn W.B., Thaler T.L., Bommarius A.S., Orville A.M. (2006). The crystal structure of NAD(P)H oxidase from *Lactobacillus*
*sanfranciscensis*: insights into the conversion of O_2_ into two water molecules by the flavoenzyme. Biochemistry.

[26] Kawakami R., Sakuraba H., Kamohara S., Goda S., Kawarabayasi Y., Ohshima T. (2004). Oxidative stress response in an anaerobic hyperthermophilic archaeon: presence of a functional peroxiredoxin in *Pyrococcus*
*horikoshii*. J. Biochem..

[27] Zheng C., Ren S., Xu J., Zhao X., Shi G., Wu J., Li J., Chen H., Bei W. (2016). Contribution of NADH oxidase to oxidative stress tolerance and virulence of *Streptococcus*
*suis* serotype 2. Virulence.

[28] Dridi B., Henry M., El Khechine A., Raoult D., Drancourt M. (2009). High prevalence of *Methanobrevibacter*
*smithii* and *Methanosphaera*
*stadtmanae* detected in the human gut using an improved DNA detection protocol. PLoS One.

[29] Million M., Tidjani Alou M., Khelaifia S., Bachar D., Lagier J.C., Dione N., Brah S., Hugon P., Lombard V., Armougom F. (2016). Increased gut redox and depletion of anaerobic and methanogenic prokaryotes in severe acute malnutrition. Sci. Rep..

[30] Hossain M.S., Dietz K.J. (2016). Tuning of redox regulatory mechanisms, reactive oxygen species and redox homeostasis under salinity stress. Front. Plant Sci..

[31] Titov D.V., Cracan V., Goodman R.P., Peng J., Grabarek Z., Mootha V.K. (2016). Complementation of mitochondrial electron transport chain by manipulation of the NAD+/NADH ratio. Science.

[32] Park J.C., Kim Y., Lee H.S. (2015). Involvement of the NADH oxidase-encoding noxA gene in oxidative stress responses in *Corynebacterium*
*glutamicum*. Appl. Microbiol. Biotechnol..

[33] Castillo-Villanueva A., Méndez S.T., Torres-Arroyo A., Reyes-Vivas H., Oria-Hernández J. (2016). Cloning, expression and characterization of recombinant, NADH oxidase from *Giardia*
*lamblia*. Protein J..

[34] Gao H., Tiwari M.K., Kang Y.C., Lee J.K. (2012). Characterization of H_2_O-forming NADH oxidase from *Streptococcus*
*pyogenes* and its application in L-rare sugar production. Bioorg. Med. Chem. Lett..

[35] Gibson C.M., Mallett T.C., Claiborne A., Caparon M.G. (2000). Contribution of NADH oxidase to aerobic metabolism of *Streptococcus*
*pyogenes*. J. Bacteriol..

[36] Kawasaki S., Ishikura J., Chiba D., Nishino T., Niimura Y. (2004). Purification and characterization of an H_2_O-forming NADH oxidase from *Clostridium*
*aminovalericum*: existence of an oxygen-detoxifying enzyme in an obligate anaerobic bacteria. Arch. Microbiol..

[37] Ward D.E., Donnelly C.J., Mullendore M.E., van der Oost J., de Vos W.M., Crane III, E.J. (2001). The NADH oxidase from *Pyrococcus*
*furiosus*. Implications for the protection of anaerobic hyperthermophiles against oxidative stress. FEBS J..

[38] Rocha-Martín J., Rivas B. d. l., Muñoz R., Guisán J.M., López-Gallego F. (2012). Rational co-immobilization of bi-enzyme cascades on porous supports and their applications in bio-redox reactions with *in situ* recycling of soluble cofactors. ChemCatChem.

[39] Beauchamp J., Gross P.G., Vieille C. (2014). Characterization of *Thermotoga*
*maritima* glycerol dehydrogenase for the enzymatic production of dihydroxyacetone. Appl. Microbiol. Biotechnol..

[40] Zhang J., Wu S., Wu J., Li Z. (2015). Enantioselective cascade biocatalysis via epoxide hydrolysis and alcohol oxidation: one-pot synthesis of (R)-α-hydroxy ketones from meso- or racemic epoxides. ACS Catal..

[41] Rocha-Martín J., Vega D., Bolivar J.M., Godoy C.A., Hidalgo A., Berenguer J., Guisán J.M., López-Gallego F. (2011). New biotechnological perspectives of a NADH oxidase variant from *Thermus*
*thermophilus* HB27 as NAD^+^-recycling enzyme. BMC Biotechnol..

[42] Zhang J., Cui Z., Chang H., Fan X., Zhao Q., Wei W. (2016). Conversion of glycerol to 1,3-dihydroxyacetone by glycerol dehydrogenase co-expressed with an NADH oxidase for cofactor regeneration. Biotechnol. Lett..

[43] Bao T., Zhang X., Rao Z., Zhao X., Zhang R., Yang T., Xu Z., Yang S. (2014). Efficient whole-cell biocatalyst for acetoin production with NAD^+^ regeneration system through homologous co-expression of 2,3-butanediol dehydrogenase and NADH oxidase in engineered *Bacillus*
*subtilis*. PLoS One.

